RETRACTED

# Everolimus ameliorates Helicobacter pylori infection-induced inflammation in gastric epithelial cells

**DOI:** 10.1080/21655979.2021.2018533

**Published:** 2022-05-04

**Authors:** Jinglei Liu, Fangxu Zhang, Zheming Zhang, Chunning Zheng

**Affiliations:** a Department of Gastrointestinal Surgery, Shandong Provincial Hospital Affiliated to shandong First Medical University, Ji’nan City, Shandong Province, China; b Department of Gastrointestinal Surgery, Clinical College of Weifang Medical University, Weifang City, Shandong Province, China

**Keywords:** Helicobacter pylori, gastritis, monocyte attachment, NF-κB, Everolimus, inflammation

## Abstract

Helicobacter pylori (*H.pylori*) infection caused by gastric mucosal inflammation plays a pivotal role in the progression of gastric diseases. The recruitment and attachment of monocytes to the gastric mucosal epithelium are a major event in the early stages of *H. pylori*-associated gastric diseases. Everolimus is a mechanistic/mammalian target of rapamycin (mTOR) inhibitor used to prevent tumor growth by inhibiting the PI3K signaling pathway. Here, we examined the pharmacological role of Everolimus against *H.pylori-*induced damage in gastric epithelial cells. Firstly, we found that Everolimus ameliorated *H.pylori-*induced oxidative stress by reducing reactive oxygen species (ROS) and malondialdehyde (MDA). Secondly, Everolimus significantly reduced the expressions of the pro-inflammatory cytokines interleukin (IL)-6, tumor necrosis factor-α (TNF-α), and IL-8. Moreover, it decreased the production of the pro-inflammatory chemokines C-X-C motif ligand 1 (CXCL1) and macrophage chemoattractant protein-1 (MCP-1). Importantly, Everolimus suppressed the induction of the adhesion molecule intracellular adhesion molecule-1 (ICAM-1) and the attachment of THP-1 monocytes to gastric epithelial AGS cells. Our data also shows that Everolimus inhibited the activation of the NF-κB signaling pathway. Therefore, we conclude that Everolimus could protect gastric epithelial cells by mitigating *H.pylori-*induced inflammatory response and the attachment of monocytes to epithelial cells.

## Introduction

Helicobacter pylori (*H. pylori*) is a gram-negative pathogenic bacterium that has been designated as a major carcinogen of human gastric cancer [1–5]. It is reported that approximately 70% of registered gastric cancer patients suffer from gastric cancer caused by *H. pylori* infection [6]. Thus, finding promising therapy for gastric diseases associated with *H. pylori* infection has increasingly attracted the interest of scientists. *H. pylori* produces a large amount of lipopolysaccharide (LPS), which is unique to Gram-negative bacteria. LPS stimulates cells to produce pro-inflammatory mediators, inducing oxidative stress and the initiation of an inflammatory response via nuclear factor kappa-B (NF-κB). In addition, activation of gastric epithelial cells caused by *H. pylori* plays a key role in the initiation and development of chronic gastritis. *H. pylori* LPS interacts with toll-like receptor (TLR)-4 and triggers the expressions of pro-inflammatory mediators, such as TNF-α, IL-6, IL-8, CXCL1, and MCP-1 [7], as well as adhesion molecules including ICAM-1, leading to the attachment of monocytes to gastric epithelial cells. Oxidative stress has been involved in aberrant epithelial damages, inflammation, and death associated with *H. pylori* infection [8,9]. *H. pylori* infection is able to increase the generation of ROS in gastric epithelial cells [10,11].

RETRACTED

Everolimus is a mechanistic/mammalian target of rapamycin (mTOR) inhibitor and is thought to inhibit tumor growth directly and indirectly by suppressing the proliferative signals of the PI3K/AKT/mTOR signaling pathway [12]. The molecular structure of Everolimus is shown in Figure 1(a). mTOR activation is critical for driving inflammatory response in an acute lung injury model [13]. mTOR inhibitors such as sirolimus have also been found to have an inhibitory effect on the expressions of pro-inflammatory chemokines such as IL-8 and MCP-1 in LPS-stimulated THP-1 and human primary monocytes via suppressing the NF-κB signaling pathway [14]. However, the effect of Everolimus on *H. pylori*-induced damage in gastric epithelial cells is unknown. The aim of our investigation is to test for the potential function of Everolimus on *H. pylori*-induced oxidative stress, inflammation, and attachment of THP-1 monocytes to gastric epithelial cells.

**Figure 1.** The effects of Everolimus on cell viability of gastric epithelial AGS cells. (a). Molecular structure of Everolimus; (b). Cells were stimulated with Everolimus at the concentrations of 0.5 2.5, 5, 25, 50, 250, 500 nM for 24 hours. Cell viability was measured using MTT assay (*, **, P < 0.05, 0.01 vs. vehicle group, N = 6).

## Material and methods

### Cell culture and treatment

AGS cells [15] and human THP-1 cells were obtained from ATCC, USA. The gastric epithelial AGS cells were cultured with Dulbecco’s modified Eagle’s medium (DMEM) (Thermo Fisher Scientific, USA) supplemented with 10% FBS, 100 U/mL penicillin, 100 mg/mL streptomycin, and L-glutamine 2 mmol/L. The medium was changed every 3 days. Before infection, the antibiotics were removed. For experimental treatment, the cells were stimulated with Helicobacter pylori (#700,392, ATCC, USA) at a bacterium/cell ratio of 500:1, followed by stimulation with Everolimus (purity ≥95%, #159,351-69-6, Sigma-Aldrich, USA) at the concentrations of 25 and 50 nM for 24 hours. THP-1 cells were grown in RPMI1640 medium (Gibco, USA) supplemented with 10% FBS, 100 U/mL penicillin, and 100 mg/mL streptomycin.

RETRACTED

### Cell viability

The effect of Everolimus on the cell viability of AGS cells was assessed using the MTT assay. Cells were plated in a 96-well plate and treated with Everolimus at the concentrations of 0, 0.5 2.5, 5, 25, 50, 250, and 500 nM for 24 hours. 20 μL of 5 mg/ml sterilized MTT (Sigma-Aldrich; USA) was added to each well. Before reading the OD value, the incubation medium was replaced with 150 μl DMSO. The absorbance was then detected with a DynaPro Plate Reader at 490 nm.

### Real-time PCR analysis

RNA was extracted from AGS cells using Fast Pure Cell RNA Isolation Kit (#RC101, Vazyme). The RNA concentration was quantified using a Nanodrop spectrometer (Thermo Fisher Scientific, USA). 2 μg RNA was transcripted to cDNA using a kit (Thermo Fisher Scientific, USA). The cDNA was subjected to qPCR with SYBR green master mix on a StepOne Plus Real-Time PCR System (Applied Biosystems). The target gene expression was normalized to GAPDH using the 2^−ΔΔCt^ method [16].

### ELISA

AGS cells were treated as described above. The supernatants were collected and stored at −80°C until further analysis. The secretions of IL-6, TNF-α, IL-8, CXCL1, MCP-1, and ICAM-1 were determined using ELISA following the product instructions. Elisa kits from R&D system were used: IL-6 (#D7050,), TNF-α (#DTA00D), IL-8 (#S8000C), CXCL1 (# SGR00B), CCL2 (# SCP00), and ICAM-1 (#SCIM00). First, 96-well cell culture plates were coated with 100 µL coating solution and incubated overnight at 4°C. After 3 washes, the plates were blocked with 200 µL blocking buffer for 1 hour at room temperature. 100 µL of standards and samples were added into designated wells and incubated for 1 hour at room temperature. After 5 washes, 100 µL of the detection antibody solution was added to each well and incubated for 2 hours at room temperature, followed by incubation with horseradish peroxidase (HRP)-linked secondary antibody for 30 minutes. 100 µL of tetramethylbenzidine (TMB) substrate solution was then added to each well and incubated for another 30 minutes. 100 µL of stop solution was then added to each well to stop the reaction. Absorbance at 450 nm was recorded to calculate the concentration of target proteins [17].

### Western blot analysis

After lysis in the RIPA buffer with protease inhibitor cocktail (Roche Diagnosis, USA) the nuclear protein was isolated using a Qproteome Nuclear Protein Kit (#37,582, QIGEN). 20 μg protein was separated on a 10% SDS-PAGE and then transferred to polyvinylidene difluoride membranes (EMD Millipore, USA). After being probed for 1 hour, the blots were incubated with the following primary antibodies from Cell signaling technology: IκBα antibody (Cat#9242), Phosphorylated IκBα antibody (Cat#2859), NF-κB p65 (Cat#3987), GAPDH (Cat#5174S), and lamin B1 (Cat#13,435), membranes were incubated with HRP Goat Anti-Rabbit (IgG) (#7074, Cell signaling Technology, USA) or Goat anti-Mouse (IgG) secondary antibody (#7076, Cell signaling Technology, USA) for 1 hour at room temperature. Blots were developed using enhanced ECL Western blotting Substrate (Thermo Fisher Scientific, USA). The blots were visualized on X-ray film with a film developer machine, and the result was analyzed using Image J software (NIH, USA) [18].

RETRACTED

### Calcein-AM staining

Attachment of THP-1 cells to gastric epithelial AGS cells was measured using calcein-AM (Cat#148,504-34-1, Abcam) staining. In brief, AGS cells were cultured in a 6-well plate until they reached ~90% confluence, and then cells were infected with Helicobacter pylori, followed by stimulation with Everolimus at the concentrations of 25 and 50 nM for 24 hours. The calcein-AM stained THP-1 cells were then added to the AGS cells and incubated for an additional 1 hour. The plates were washed thoroughly to remove the unattached cells and then observed under a fluorescence microscope (Zeiss Autoplan2).

### Dihydroethidium (DHE) assay

Intracellular ROS in AGS cells was measured using DHE staining. After treatment, cells were incubated with 5 μM DHE and incubated for 15 minutes at 37°C in darkness. Fluorescent signals were visualized using a fluorescent microscope. The level of ROS was quantitated using Image J software.

### Malondialdehyde (MDA) assay

MDA concentration in AGS cells was examined using a kit (Calbiochem, USA). The cell lysate was mixed with N-methyl-2-phenylindole in acetonitrile in the ratio of 1:3, followed by adding 1% HCl and incubated at 45°C for 1 hour. Absorbance was recorded at 586 to index MDA concentration.

### Luciferase activity of NF-κB

Cells were co-transfected with luciferase reporter plasmid pNF-κB-Luc (0.1 μg) and pRL-TK plasmid (0.05 μg) (Promega, USA). 12 hours later, cells were infected with Helicobacter pylori, followed by stimulation with Everolimus at the concentrations of 25 and 50 nM. Firefly luciferase and Renilla luciferase activities were determined using the Dual-luciferase reporter assay system (Promega, USA). Renilla luciferase activity was used as a normalization control.

### Statistical analysis

All results were displayed as Mean ± standard deviation (S.D.). Statistical analysis was performed by Prism 7.05 (GraphPad, USA). Comparisons were performed using analysis of variance (ANOVA) with Bonferroni’s post-hoc test. A P-value less than 0.05 was considered as a significant difference.

RETRACTED

### Results

In order to investigate the effects of Everolimus on *H. pylori*-challenged gastric epithelial AGS cells, we tested several important factors. First, we investigated the potential benefits of Everolimus on oxidative stress and the expression of pro-inflammatory cytokines. Then we investigated the effects of Everolimus on the attachment of THP-1 by inhibiting the expression of adhesion molecules such as ICAM-1. Importantly, we further clarified the involvement of NF-κB in this inflammatory response.

### The effects of Everolimus on the cell viability of gastric epithelial AGS cells

First, we assessed the cytotoxicity of Everolimus in AGS cells. When the concentration of Everolimus was lower than 50 nM, the cell viability was not affected (Figure 1(b)). However, when the concentration of Everolimus was higher than 50 nM, the cell viability of gastric epithelial cells was reduced significantly to 91% (250 nM of Everolimus) and 83% (500 nM of Everolimus). Therefore, 25 and 50 nM Everolimus were used in this study.

### *Everolimus ameliorates* H. pylori-*induced oxidative stress*

To clarify the effect of Everolimus on *H. pylori-*induced oxidative stress in gastric epithelial cells, the generation of ROS and production of MDA were measured. As shown in Figure 2(a), the generation of ROS was remarkably elevated to 3.3- fold by *H. pylori* only and decreased to 2.4- and 1.7- fold by 25 and 50 nM of Everolimus, respectively. Similarly, as shown in Figure 2(b), the production of MDA was inhibited to 2.2- and 1.6- fold by the same doses of Everolimus, respectively, compared to a 2.9- fold increase stimulated by *H. pylori*. These results indicate the anti-oxidative effect of Everolimus on *H. pylori-*challenged gastric epithelial cells.

**Figure 2.** Everolimus ameliorates Helicobacter pylori-induced oxidative stress. Cells were infected with Helicobacter pylori at a bacterium/cell ratio of 500:1, followed by stimulation with Everolimus at the concentrations of 25 and 50 nM for 24 hours. (a). Intracellular levels of ROS; Scale bar, 100 μm; (b). Levels of intracellular MDA were measured (####, P < 0.0001 vs. vehicle group;$, P < 0.01, 0.001 vs. Helicobacter pylori group, N = 5).

### *Everolimus inhibits* H. pylori-*induced expression of pro-inflammatory mediators*

As pro-inflammatory cytokines play a critical role in gastric inflammation, we examined the effect of Everolimus on *H. pylori-induced* expressions of IL-6, TNF-α, and IL-8. The mRNA level of IL-6 increased approximately by 3.9- fold after exposure to *H. pylori* alone, but 25 and 50 nM Everolimus reduced it to approximately 2.7- and 1.8- fold, respectively (Figure 3(a)). The same doses of Everolimus decreased the mRNA level of TNF-α to 2.0- and 1.5- fold, respectively, compared to a 2.6- fold increase from exposure to *H. pylori* (Figure 3(b)). The mRNA level of IL-8 was reduced to 2.4- and 1.6- fold by Everolimus, respectively, compared to a 3.3-fold increase induced by *H. pylori* (Figure 3(c)). Similarly, 25 and 50 nM Everolimus significantly inhibited the secretions of IL-6, TNF-α, and IL-8 at their protein levels (Figure 3(d-f)).

RETRACTED

**Figure 3.** Everolimus inhibits Helicobacter pylori-induced expression and secretions of IL-6, TNF-α, and IL-8. (a-c). mRNA of IL-6, TNF-α, IL-8; (d). Secretions of IL-6; (e). Secretions of TNF-α; (f). Secretions of IL-8 (####, P < 0.0001 vs. vehicle group;$, P < 0.01, 0.001 vs. Helicobacter pylori group, N = 5).

We then tested for the role of Everolimus on the expressions and secretions of CXCL1 and MCP-1, which are important chemokines in gastric epithelial cells. Our results show that 25 and 50 nM Everolimus downregulated the expression of CXCL1 to 2.9- and 2.1- fold at the mRNA level, respectively, compared to a 4.2- fold increase from exposure to *H. pylori* only (Figure 4(a)). Similarly, *H. pylori-*stimulation increased the mRNA level of MCP-1 to 3.4- fold, which was dose-responsively decreased to 2.5- and 1.6- fold by the two doses of Everolimus (Figure 4(b)). Additionally, Everolimus significantly suppressed the secretions of CXCL1 and MCP-1 at the protein levels (Figure 4(c-d)).

**Figure 4.** Everolimus suppresses Helicobacter pylori-induced expressions and secretions of CXCL1 and MCP-1. (a-b). mRNA of CXCL1and MCP-1; (c). Secretion of CXCL1; (d). Secretion of MCP-1 (####, P < 0.0001 vs. vehicle group; $, P < 0.01, 0.001 vs. Helicobacter pylori group, N = 5).

### *Everolimus suppresses* H. pylori-induced *expression of ICAM-1 and the attachment of THP-1 cells to gastric epithelial AGS cells.*

Next, we assessed the effects of Everolimus on the expression of ICAM-1, an important adhesion molecule that mediates the attachment of monocytes to gastric epithelial cells. *H. pylori* increased the expression of ICAM-1 to 3.8- fold at the mRNA level (Figure 5(a)), which was downregulated to 2.7- and 2.1- fold by 25 and 50 nM Everolimus, respectively. Similarly, the same doses of Everolimus decreased the protein level of ICAM to 267.6 and 158.7 pg/mL, initially increased to 426.5 pg/mL by exposure to *H. pylori* only (Figure 5(b)).

**Figure 5.** Everolimus suppresses Helicobacter pylori-induced expression of ICAM-1 in gastric epithelial AGS cells. (a). mRNA of ICAM-1; (b). Secretion of ICAM-1 (####, P < 0.0001 vs. vehicle group; $, P < 0.01, 0.001 vs. Helicobacter pylori group, N = 5).

RETRACTED

We then investigated the effect of Everolimus on *H. pylori-induced* attachment of THP-1 cells to gastric epithelial AGS cells. The attachment of THP-1 cells was increased 4.2- fold by *H. pylori-*stimulation but reduced to 2.7- and 1.9- fold by 25 and 50 nM Everolimus, respectively (Figure 6(a)). To clarify whether the effects of Everolimus on *H. pylori-induced* attachment of THP-1 cells to gastric epithelial AGS cells are dependent on or independent of mTOR inhibition, another mTOR inhibitor, Rapamycin was used. Interestingly, results in Figure 6(b) indicate that treatment with Rapamycin did not have a significant impact on *H. pylori-*induced attachment of THP-1 cells to gastric epithelial AGS cells, suggesting that the effect of Everolimus might be independent of the inhibition of mTOR.

**Figure 6.** Everolimus but not Rapamycin suppresses Helicobacter pylori-induced attachment of THP-1 cells to gastric epithelial AGS cells. (a). Cells were infected with Helicobacter pylori at a bacterium/cell ratio of 500:1, followed by stimulation with Everolimus at the concentrations of 25 and 50 nM for 24 hours. Attachment of THP-1 cells to gastric epithelial AGS cells was measured using calcein-AM staining. (b). Cells were infected with Helicobacter pylori at a bacterium/cell ratio of 500:1, followed by stimulation with Rapamycin at the concentrations of 25 and 50 nM for 24 hours. Attachment of THP-1 cells to gastric epithelial AGS cells was measured using calcein-AM staining. Scale bar, 100 μm (####, P < 0.0001 vs. vehicle group; $, P < 0.01, 0.001 vs. Helicobacter pylori group, N = 5).

### *Everolimus prevents* H. pylori-induced *activation of the IκBα/NF-κB signaling pathway*

The results in Figure 7 indicate that *H. pylori-*stimulation increased the phosphorylation of IκBα to 3.4- fold, which was decreased to 2.4- and 1.6- fold by 25 and 50 nM Everolimus, respectively. Then, we found that the same doses of Everolimus rescued the total IκBα to 73% and 91%, compared to a 53% decrease stimulated by *H.pylori*. Our data shows that *H.pylori-*stimulation significantly increased the nuclear levels of p65 to 3.6- fold, which was later downregulated to 2.7- and 1.6- fold by 25 and 50 nM Everolimus, respectively (Figure 8(a)). The luciferase activity of NF-κB was reduced to 271.2- and 193.3- fold by the same doses of Everolimus, compared to a 365.6-fold increase induced by *H.pylori* (Figure 8(b)).

**Figure 7.** Everolimus suppresses Helicobacter pylori-induced phosphorylation and degradation of IκBα. Cells were infected with Helicobacter pylori, followed by stimulation with Everolimus at the concentrations of 25 and 50 nM for 6 hours. Phosphorylated and total IκBα were measured (####, P < 0.0001 vs. vehicle group;$, P < 0.01, 0.001 vs. Helicobacter pylori group, N = 4).

RETRACTED

**Figure 8.** Everolimus suppresses Helicobacter pylori-induced activation of NF-κB. Cells were infected with Helicobacter pylori, followed by stimulation with Everolimus at the concentrations of 25 and 50 nM for 6 hours. (a). Nuclear levels of NF-κB p65; (b). Luciferase activity of NF-κB (####, P < 0.0001 vs. vehicle group;$, P < 0.01, 0.001 vs. Helicobacter pylori group, N = 4).

## Discussion

Oxidative stress, inflammation, and monocyte adhesion play a pivotal role in the development of *H.pylori* infection-associated gastric diseases. Here, we examined the protective effects of Everolimus on *H.pylori*-stimulated gastric epithelial cells. Previous studies have demonstrated that *H.pylori* infection remarkably reduced the expressions of antioxidant enzymes such as SOD and reduced GSH in human gastric epithelial cells [19,20]. Our results show that *H.pylori* infection significantly increased the expressions of ROS and MDA. It has been reported that the overproduction of ROS in *H.pylori-*stimulated gastric epithelial cells depends on NADPH oxidase, which could be directly activated by *H.pylori* infection [21]. The excessive generation of ROS plays an important role in cellular oxidative stress mechanisms of chronic gastritis through the induction of MDA and cell apoptosis [22,23]. Furthermore, previous research indicates that ROS can regulate the mTOR-related signaling pathway to be involved in cell autophagy [24]. mTOR inhibition has displayed an inhibitory capacity in the generation of ROS [25]. In this study, we show new evidence that Everolimus could alleviate oxidative stress by inhibiting *H.pylori*-induced generation of ROS and the production of MDA.

Monocyte attachment has been reported to play a vital role in *H.pylori-*associated gastric diseases and has been considered the main treatment target. As our results have shown that Everolimus significantly suppressed the attachment of THP-1 cells to gastric epithelial cells, we believe that it could be a potential therapeutic agent. Pro-inflammatory cytokines and chemokines are major factors in the progression of *H.pylori-*associated gastric diseases. TNF-α is a well-known cytokine for its role in initiating the inflammatory cascade to trigger the production of various other inflammatory factors and induction of cell death [26]. IL-6 and IL-8 are considered key elements involved in the progression of gastritis because they have broad biological effects on mononuclear cells [27]. Furthermore, IL-8, CXCL1, and MCP-1 are responsible for monocyte migration to the sites of infection in *H.pylori-*associated gastric diseases [28–30]. *H.pylori* infection highly increased the expressions of IL-8, CXCL1, and MCP-1 in gastric mucosa tissues of patients [31–33]. In our study, we found that Everolimus greatly inhibited the increased levels of these pro-inflammatory regulators induced by *H.pylori*. ICAM-1 is significantly upregulated at sites of inflammation in *H.pylori-*stimulated gastric epithelial cells, indicating the important role of ICAM-1 in *H.pylori*-related gastric diseases. Our findings show that Everolimus robustly reduced the expression of ICAM-1, implying its beneficial effect against *H.pylori-*induced immune attachment to epithelial cells. NF-κB is activated during *H. pylori* infection in various types of cells [34,35]. The expressions of IL-6, TNF-α, IL-8, CXCL1, MCP-1, and ICAM-1 in *H.pylori-*stimulated gastric epithelial cells are mediated by NF-κB [36–38]. *H.pylori* activates NF-κB by phosphorylating and degrading IκBα, promoting NF-κB p65 to translocate into the nucleus and bind to the promoter of DNA sequences. Inhibition of the NF-κB signaling pathway could be impactful for protecting against gastric diseases [32]. Additionally, the NF-κB system has been found to be deregulated in gastric cancer and recommended for therapeutic targeting. Here, we demonstrate that Everolimus prevented the activation of NF-κB by inhibiting the phosphorylation and degradation of IκBα, suggesting a promising therapeutic effect of Everolimus in *H. pylori*-associated gastric diseases. In recent decades, antibiotic treatment is considered a therapeutic strategy against *H. pylori*. Clarithromycin, Metronidazole, and Tetracycline have been widely used for the treatment of *H. pylori*-associated diseases. In fact, these antimicrobials have been shown to exert powerful benefits in *H. pylori*-associated diseases. However, due to the misuse of antibiotics, antibiotic resistance has become an increasing problem [39]. Compared with traditional antibiotic treatment, Everolimus prevents inflammation in *H. pylori*-associated disease by regulating signaling pathways such as NF-κB, thereby avoiding antibiotic resistance.

RETRACTED

The mechanism of inflammatory response in gastric diseases is still complex. Previous studies have shown that activated mTOR could promote activation of the NF-κB signaling pathway in neuro-inflammation of Parkinson’s disease and in an *in vivo* obstructive sleep apnea (OSA) model [40,41]. Dan *et al*. (2008) further clarified the underlying mechanism by which mTOR regulates the activation of NF-κB [42]. These findings indicate that Everolimus, an mTOR inhibitor, may exert its anti-inflammatory benefits through the mTOR/ NF-κB signaling pathway. However, it is also possible that Everolimus directly regulates the NF-κB signaling pathway. The pharmacological mechanisms of Everolimus are limited. Interestingly, the activation of extracellular signal-regulated kinase (ERK) by Everolimus has been associated with its limited efficacy in gastric cancer. The combined inhibition with Everolimus and trametinib can overcome resistance by specifically inhibiting ERK and regulating ERK-mediated Bcl-2 family proteins in gastric cancer cells [43]. Our preliminary experiments (Figure 1b) indicate that 25 and 50 nM Everolimus are both optimal concentrations used for the treatment in AGS cells, which is relevant to the doses used in clinics [44]. In our future work, we will further study the effects of Everolimus on *H. pylori*-associated gastric diseases, to reveal the full picture of the underlying mechanism involved in gastric diseases.

## Conclusion

In summary, our study provides new evidence that Everolimus suppresses oxidative stress and monocyte attachment in *H.pylori-*stimulated gastric epithelial cells, indicating a potential protective effect of Everolimus on *H.pylori*-induced gastric diseases. However, the mechanisms of *H.pylori* infection-related gastric diseases are still complicated, more research is required to further elucidate the benefits of Everolimus.

## Availability of Data Materials

The data that support the findings of this study are available from the corresponding author upon reasonable request.

## References

[1] Correa P. Human gastric carcinogenesis: a multistep and multifactorial process-First American cancer society award lecture on cancer epidemiology and prevention. Cancer Res. 1992;52:6735–6740.1458460

[2] Bj M, Jr W. Unidentifified curved bacilli in the stomach of patients with gastritis and peptic ulceration. Lancet. 1984;1:1311–1315.614502310.1016/s0140-6736(84)91816-6

[3] Uemura N, Okamoto S, Yamamoto S, et al. Helicobacter pylori infection and the development of gastric cancer. N Engl J Med. 2001;345:784–789.1155629710.1056/NEJMoa001999

[4] Ito N, Tsujimoto H, Ueno H, et al. Helicobacter pylori-mediated immunity and signaling transduction in gastric cancer. J Clin Med. 2020;9:3699.10.3390/jcm9113699PMC769875533217986

[5] Parsonnet J, Friedman GD, Vandersteen DP, et al. Helicobacter pylori infection and the risk of gastric carcinoma. N Engl J Med. 1991;325:1127–1131.189102010.1056/NEJM199110173251603

RETRACTED

[6] Bray F, Ferlay J, Soerjomataram I, et al. Global cancer statistics 2018: GLOBOCAN estimates of incidence and mortality worldwide for 36 cancers in 185 countries. CA Cancer J Clin. 2018;68:394.3020759310.3322/caac.21492

[7] Sugimoto M, Furuta T, Yamaoka Y. Influence of inflammatory cytokine polymorphisms on eradication rates of Helicobacter pylori. J Gastroenterol Hepatol. 2009;24:1725–1732.2013695910.1111/j.1440-1746.2009.06047.xPMC3128255

[8] Clement MV, Pervaiz S. Reactive oxygen intermediates regulate cellular response to apoptotic stimuli: a hypothesis. Free Radic Res. 1999;30:247–252.1023080310.1080/10715769900300271

[9] Baik SC, Youn HS, Chung MH, et al. Increased oxidative DNA damage in Helicobacter pylori-infected human gastric mucosa. Cancer Res. 1996;56:1279–1282.8640814

[10] Sobalo GM, Schorah CJ, Shires S, et al. Effect of eradication of Helicobacter pylori on gastric juice ascorbic acid concentrations. Gut. 1993;34:1038–1041.817494910.1136/gut.34.8.1038PMC1374349

[11] Nagata K, Yu H, Nishikawa M, et al. Helicobacter pylori generates superoxide radicals and modulates nitric oxide metabolism. J Biol Chem. 1998;273:14071–14073.960390210.1074/jbc.273.23.14071

[12] Du L, Li X, Zhen L, et al. Everolimus inhibits breast cancer cell growth through PI3K/AKT/mTOR signaling pathway. Mol Med Rep. 2018;17(5):7163–7169.2956888310.3892/mmr.2018.8769PMC5928673

[13] Ma C, Zhu L, Wang J, et al. Anti-inflammatory effects of water extract of Taraxacum mongolicum hand-Mazz on lipopolysaccharide -induced inflammation in acute lung injury by suppressing PI3K/Akt/mTOR signaling pathway. J Ethnopharmacol. 2015;168:349–355.2586195410.1016/j.jep.2015.03.068

[14] Lin HY, Chang KT, Hung CC, et al. Effects of the mTOR inhibitor rapamycin on monocyte-secreted chemokines. BMC Immunol. 2014;15:37.2525797610.1186/s12865-014-0037-0PMC4189728

[15] Morey P, Pfannkuch L, Pang E, et al. Helicobacter pylori depletes cholesterol in gastric glands to prevent interferon gamma signaling and escape the inflammatory response. Gastroenterology. 2018;154(5):1391–1404.e9.2927345010.1053/j.gastro.2017.12.008

[16] Wen L, Cheng FJ. Circular RNA circCRKL inhibits the proliferation of acute myeloid leukemia cells via the miR-196a-5p/miR-196b-5p/p27 axis. Bioengineered. 2021;12(1):7704–7713.3461787610.1080/21655979.2021.1982310PMC8806729

[17] Lv YL, Zhang JH, Wang CY. Self-assembled chitosan nanoparticles for intranasal delivery of recombinant protein interleukin-17 receptor C (IL-17RC): preparation and evaluation in asthma mice. Bioengineered. 2021;12(1):3029–3039.3418076410.1080/21655979.2021.1940622PMC8806589

[18] Zhou XY, Wang ZL, Xu BC, et al. Long non-coding RNA NORAD protects against cerebral ischemia/reperfusion injury induced brain damage, cell apoptosis, oxidative stress and inflammation by regulating miR-30a-5p/YWHAG. Bioengineered. 2021;12(2):9174–9188.3470997210.1080/21655979.2021.1995115PMC8810080

RETRACTED

[19] Beil W, Obst B, Sewing KF, et al. Helicobacter pylori reduces intracellular glutathione in gastric epithelial cells. Dig Dis Sci. 2000;45:1769–1773.1105231810.1023/a:1005530227603

[20] Li S, Wu D, Cao M, et al. Effects of choline supplementation on liver biology, gut microbiota, and inflammation in Helicobacter pylori-infected mice. Life Sci. 2020;259:118200.3275862110.1016/j.lfs.2020.118200

[21] Kim SH, Lim JW, Kim H. Astaxanthin inhibits mitochondrial dysfunction and interleukin-8 expression in helicobacter pylori-infected gastric epithelial cells. Nutrients. 2018;10:1320.10.3390/nu10091320PMC616477030231525

[22] Slomiany A, Piotrowski E, Piotrowski J, et al. Impact of ethanol on innate protection of gastric mucosal epithelial surfaces and the risk of injury. J Physiol Pharmacol. 2000;51:433–447.11016863

[23] Shindo Y, Konagaya M, Harasawa S, et al. The role of histamine in ethanol-induced gastric mucosal injury in the rat. Tokai J Exp Clin Med. 1997;22:59–64.9608632

[24] Zhou Y, Wang Y, Zhou W, et al. YAP promotes multi-drug resistance and inhibits autophagy-related cell death in hepatocellular carcinoma via the RAC1-ROS-mTOR pathway. Cancer Cell Int. 2019;19:179.3133798610.1186/s12935-019-0898-7PMC6626386

[25] Kida T, Oku H, Osuka S, et al. Hyperglycemia-induced VEGF and ROS production in retinal cells is inhibited by the mTOR inhibitor, Rapamycin. Sci Rep. 2021;11(1):1885.3347932810.1038/s41598-021-81482-3PMC7820225

[26] Shu ZG, Angela F, Messmer B, et al. Role of A20 in cIAP-2 protection against tumor necrosis factor α (TNF-α)-mediated apoptosis in endothelial cells. Int J Mol Sci. 2014;15:3816–3833.2459524210.3390/ijms15033816PMC3975369

[27] Akira S, Hirano T, Taga T. Biology of multifocal cytokines: IL6 and related molecules (IL1 and TNF). FASEB J. 1990;4:2860–2867.2199284

[28] Soderquist B, Kallman J, Holmberg H, et al. Secretion of IL-6, IL-8 and G-CSF by human endothelial cells in vitro in response to Staphylococcus aureus and staphylococcal exotoxins. APMIS. 1998;106:1157–1164.10052724

[29] Tekstra JH, Beekhuizen JS, Van De Gevel IJ, et al. Infection of human endothelial cells with Staphylococcus areus induces the production of monocyte chemotactic protein-1 (MCP-1) and monocyte chemotaxis. Clin Exp Immunol. 1999;117:489–495.1046905210.1046/j.1365-2249.1999.01002.xPMC1905370

[30] Innocenti M, Thoreson AC, Ferrero RL, et al. Helicobacter pylori-induced activation of human endothelial cells. Infect Immun. 2002;70:4581–4590.1211797110.1128/IAI.70.8.4581-4590.2002PMC128191

RETRACTED

[31] Watanabe N, Shimada T, Ohtsuka Y, et al. Proinflammatory cytokines and Helicobacter pylori stimulate CC-chemokine expression in gastric epithelial cells. J Physiol Pharmacol. 1997;48:405–413.9376623

[32] Shimoyama T, Everett SM, Dixon MF, et al. Chemokine mRNA expression in gastric mucosa is associated with Helicobacter pylori cagA positivity and severity of gastritis. J Clin Pathol. 1998;51:765–770.1002334010.1136/jcp.51.10.765PMC500932

[33] Jung HC, Kim JM, Song IS, et al. Helicobacter pylori induces an array of pro-inflammatory cytokines in human gastric epithelial cells: quantification of mRNA for interleukin –8-1 alpha/beta, granulocyte–macrophage colony-stimulating factor, monocyte chemoat tractant protein-1 and tumor necrosis factor-alpha. J Gastroenterol Hepatol. 1997;12:473–480.925723610.1111/j.1440-1746.1997.tb00469.x

[34] Aihara M, Tsuchimoto D, Takizawa H, et al. Mechanisms involved in Helicobacter pylori-induced interleukin-8 production by a gastric cancer cell line, MKN45. Infect Immun. 1997;65:3218–3224.923477810.1128/iai.65.8.3218-3224.1997PMC175455

[35] Keates S, Hitti YS, Upton M, et al. Helicobacter pylori infection activates NF-kappa B in gastric epithelial cells. Gastroenterology. 1997;113:1099–1109.932250410.1053/gast.1997.v113.pm9322504

[36] Mori N, Wada A, Hirayama T, et al. Activation of intercellular adhesion molecule 1 expression by Helicobacter pylori is regulated by NF-kappaB in gastric epithelial cancer cells. Infect Immun. 2011;79:542.2117793110.1128/IAI.01065-10PMC3019916

[37] Sharma SA, Tummuru MK, Blaser MJ, et al. Activation of IL-8 gene expression by helicobacter pylori is regulated by transcription factor nuclear factor -kappa B in gastric epithelial cells. J Immunol. 1998;160:2401–2407.9498783

[38] Bagheri N, Azadegan-Dehkordi F, Shirzad H, et al. The biological functions of il-17 in different clinical expressions of helicobacter pylori-infection. Microb Pathog. 2015;81:33–38.2577377110.1016/j.micpath.2015.03.010

[39] Tshibangu-Kabamba E, Yamaoka Y. Helicobacter pylori infection and antibiotic resistance - from biology to clinical implications. Nat Rev Gastroenterol Hepatol. 2021 Sep;18(9):613–629. doi:10.1038/s41575-021-00449-x.34002081

[40] Rasheed M, Liang J, Wang C, et al. Epigenetic regulation of neuroinflammation in Parkinson’s disease. Int J Mol Sci. 2021;22:4956.3406694910.3390/ijms22094956PMC8125491

[41] Zhang CQ, Yi S, Chen BB, et al. mTOR/NF-κB signaling pathway protects hippocampal neurons from injury induced by intermittent hypoxia in rats. Int J Neurosci. 2021;131(10):994–1003. doi:10.1080/00207454.2020.1766460.32378972

RETRACTED

[42] Hc D, Mj C, Pc C, et al. Akt-dependent regulation of NF-kappaB is controlled by mTOR and Raptor in association with IKK. Genes Dev. 2008;22:1490–1500.1851964110.1101/gad.1662308PMC2418585

[43] Liu HF, Yao Y, Zhang J, et al. MEK inhibition overcomes everolimus resistance in gastric cancer. Cancer Chemother Pharmacol. 2020;85(6):1079–1087.3244489710.1007/s00280-020-04078-0

[44] Nölting S, Garcia E, Alusi G, et al. Combined blockade of signalling pathways shows marked anti-tumour potential in phaeochromocytoma cell lines. J Mol Endocrinol. 2012;49(2):79–96.2271516310.1530/JME-12-0028PMC4714579

